# Healthism online: ‘What I eat in a day’ vlogs before and during COVID-19 restrictions

**DOI:** 10.1016/j.heliyon.2023.e23623

**Published:** 2023-12-13

**Authors:** Elisa Eltink, Christian Bröer

**Affiliations:** a Communication, Health and Life Sciences, Wageningen University, PO Box 8130, 6700 EW, Wageningen, the Netherlands; b Department of Sociology, University of Amsterdam, Nieuwe Achtergracht 166, 1018 WV, Amsterdam, the Netherlands

**Keywords:** COVID-19, Social sciences, Healthism, Health, Social Media, Lifestyle, Diet, Vlogs, overweight

## Abstract

**Objective and setting:**

The COVID-19 pandemic and its restrictions coincide with an increase in body weight and changes in health-related habits worldwide. This study focusses on the way health-related habits are portrayed online in digital food cultures. The study aims to investigate if and how the content of high-profile Dutch ‘What I eat in a day’ vlogs has changed during the first period of COVID-19 restrictions. We approach changes in digital food culture through the concept of ‘healthism’ and see vloggers as cultural intermediaries.

**Design and participants:**

We collected the most watched vlogs of almost all high-profile Dutch influencers pre-post corona and analyzed these in a mixed method approach by using summative and thematic content analysis.

**Results:**

Pre-COVID vlogs highlight an explicit consciousness of energy balance-related behavior, focusing on calorie counting, avoidance of unhealthy food and the use of tracking apps. In vlogs uploaded in 2020, these themes are less present. Instead, intuitive eating and listening to one’s body are more central themes within the vlogs.

**Conclusions:**

We consider the shift towards intuitive eating as another variant of “wellness diets” rather than a shift away from dieting, furthered by COVID-19 restrictions. The core values of health and self-regulation are upheld within the shift towards intuitive eating. Yet, we nuance the broad claims of healthism in biopolitics and point to relevant cultural changes within foodscapes.

## 1 Introduction

The COVID-19 pandemic and its restrictions coincide with a rise in body weight [[1], [2], [3], [4]]. A 2021 study in 30 different countries has shown that almost one-third of the world population has gained weight during the pandemic [5]. Simultaneously, eating, drinking, supplement intake [6] and physical activity patterns changed during the pandemic, albeit research showed seemingly diverse results. Longitudinal studies [7] demonstrate an increase in snacking, eating sweets and ultra-processed food in addition to drinking more alcohol on average. At the same time, sub-groups report stable habits or even improved diets [8]. Focusing on alcohol consumption, an EU-wide meta-analysis showed both increase, decrease and stability, the latter particularly among heavy drinkers [9]. When it comes to physical activity, the patterns are similarly diverse [10], showing less but also stable activity patterns. Across different studies, we see that changes during the pandemic depend on gender, age, health status, prior habits, education and country context at least. We thus plea for a more nuanced, country-level analytical lens. What the abovementioned studies do not focus on are changes in media reporting about food and exercise during COVID-19 restrictions, which we address here. Looking at body weight from a system perspective instead of focusing on individual behavior [11], we see that media play an important role in the lives of adolescent in relation to body weight and food intake [12]. By looking at media reporting before and during restrictions, we aim to take a first step towards understanding the relevance of cultural changes for food practices and health during COVID-19.

Changes in weight and weight related practices might indicate a change in food-cultures. In this study we focus on the way eating habits are promoted in “digital food cultures” [13,14]. Online, traditional foodscape shifted towards a ‘mediated foodscape’ [15] which calls for a broader engagement with complex and diverse media formats [16]. Food media has the power to *frame* and *mediate* what foodscapes could and should be. Food media communicates food instructions via recipes and simultaneously projects powerful images of what constitutes a good meal, desirable looks and a good life in general. Because of this, food media and the mediatized foodscapes contribute to the biopolitics of everyday life [15].

In this article, we are particularly focusing on the role of healthism – individualized health as dominant ideology – in mediated foodscapes [17]. Crawford early on argued that health has become a matter of individual responsibility and a core striving of modern life. Epstein and Timmermans [18] in their study in the United States, found a shift and diversification of authority in the landscape of medicine and health. In this new landscape, alternative ways of healing and new forms of self-care and self-monitoring are more prominent compared to the traditional practices of biomedicine. In this sense, the authority of biomedicine in the United States shifted to cultural authorities outside of the medical profession. Especially in recent years, the achievement of health and wellness has become both a moral imperative and a source of moral judgment about how to look, live or behave [18].

In our study, this social effort to gain control over health becomes manifested in both omnipresent personal attempts at ‘body control’ and widespread ‘health claims’. Health claims are often made about nutritional values or expected effects of products (e.g. I take lemon water because it helps with digestion). As Crawford [17] argues that health is a moral discourse that confirms shared beliefs and cultural values, the use of health claims should similarly be perceived as such a kind of moral discourse. Health claims are often made to strive to change the shape of the body. Therefore, body control entails the individualized moral obligation that people are responsible for the shape of their bodies. In the area of food and weight, this pushes people to lose weight by exercising and being conscious of their food intake and nutritional values. This way of approaching food shows similarities with orthorexia [19], since people with orthorexia strive to ‘eat right’, by focusing on ‘pure’ and ‘clean’ products, upholding healthism as ideology.

Using this lens of healthism, Delaney & McCarthy [20] study how: *moral talk about food and eating reflected a complicated relationship between food and pleasure* (p.108) where food has often been broken down into the moral binaries of ‘good’/‘bad and ‘healthy’ ‘unhealthy’. Braun and Carruthers [14] explain how most contemporary diets, like paleo, keto or sugar-free diets, reflect these binaries and that restriction and elimination is the uniting factors of all diets. In line with the concept of healthism, Braun and Carruthers term these diets as ‘wellness diets’, *because they evoke an ideal of optimal health, achievable through the correct diet, and because they often merge into other aspects of living* (p. 83).

Contemporary discourses on health are observable in the proliferation of ‘food influencers’ and bloggers on social media. In *digital food cultures,* Lupton [13] describes how social media influencers play an important role in drawing attention to food cultures and trends whereby these so–called lifestyle influencers focus on aspects of daily life practices like dieting, food prepping and cooking. A rising scene in this world of influencers are ‘What I eat in a day’ vlogs, where ‘vloggers’ distribute their eating, cooking, and sporting habits to a wide audience on YouTube [see [21] for physical exercise videos]. Using Crawford’s concept of healthism, we see that these vlogs are composed of both individualizing advice on body control and health claims. As youth and young adults increasingly approach social media as a source of medical information [22], the depicted lifestyles of ‘What I eat in a day’ vloggers could be appropriated by their followers [23]. In the words of Bourdieu [24], food influencers can therefore be perceived as ‘cultural intermediaries’ as they are ultimately “sellers of symbolic goods and services who sell themselves as models and as guarantors of the value of their products” (p. 365). Social media platforms disrupted traditional health information authority and expertise and shifted engagement with the various sources of ‘advice’ being available on the internet. Such digital cultures reinforce the message that people areself-directing agents who are responsible for their own health [14].

This research has focused on the content of ‘What I eat in a day’ vlogs to see if the messages constructed by high profile vloggers in the Netherlands have changed during the first period of COVID-19 restrictions. We do not claim causality, since vloggers are as much drivers as symptoms of trends in eating and dieting. Instead, this article tries to interpret the role of ‘What I eat in a day’ vloggers as cultural intermediaries in the rise of novel eating practices. Hence, the research question has been “*How do ‘What I eat in a day’ vlogs before and during the first months of COVID-19 differ from each other concerning body control and health claims and how can we interpret these changes from the perspective of healthism and digital food cultures?*”.

## 2 Methods

The research question is answered through a **quantitative** and **qualitative** content analysis approach of ‘What I eat in a day’ vlogs on YouTube. In 2019 and 2020 we have included almost all videos available on YouTube in the following way: We have first identified all Dutch speaking “What I eat in a day” vloggers in 2019 and 2020. For 2019 we included all vloggers and for 2020 almost all of them. For both years we included the most watched video of each vlogger. Together these vlogs have been watched 812.902 times at the moment of data collection. Our sample thus covers the largest part of Dutch “What I eat in a day vlogs” in 2019 and 2020.

The videos uploaded in 2019 are approached as comparative cases for the potential effect of COVID-19. We have chosen to analyze Dutch language vloggers because of the Dutch descent of the researchers, aiding to enhance the interpretation of cultural practices. The data collection eventually led to a total of 37 videos: 16 videos from 2019 and 21 from 2020. The cases were analyzed by using summative content analysis [25,26] and thematic content analysis using a coding logbook which is commonly used in these kind of studies to track the process and decisions of manual coding.

For the **quantitative** content analysis, an inductively constructed codebook served as a guideline for further analysis. The codes were inductively derived by watching Dutch ‘What I eat in a day’ vlogs. All expressions or behaviors that were deemed relevant were coded literally or thematically for manifest meanings (e.g: mentioning protein value). After saturation was reached, meaning no relevant codes or themes were found within the videos, the codes were clustered into seven thematic categories.

Category one entailed health and product claims created by the concerned vloggers (e.g: this product contains a lot of protein), category two consisted of marketing and lifestyles, like showing bought products. The third category consisted of expressions and behaviors of body control, i.e. wanting to lose weight. The fourth category was formed based on statements about COVID-19 expressed by the vloggers. Talking about different diet types, like the keto diet or intermitted fasting, were clustered in category five. The sixth category consisted of health behaviors related to emotions, like emotional eating or eating to ‘feel good’. The seventh and last category was about taste and esthetics, i.e. consuming foods because they look good on video. Besides the seven categories, frequently mentioned food products such as ginger tea, lemon water and avocado toast were taken into the codebook as well. Subsequently, frequencies of codes were collected in a SPSS database and codes were combined to form an index based on thematic congruence. This allowed for a more conceptual analysis with T-tests to compare the averages of the mentioned themes.

The quantitative part gave insight in the manifest meanings of the food vlogs. To deepen this knowledge and to shed a light on the latent meanings of the food vlogs, a **qualitative** thematic analysis was performed, following the six phases of thematic analysis [26]. Phase one consisted of getting familiar with the data. In this phase, relevant elements in the vlogs were transcribed and collected in a document. The second step contained coding. Here, the transcribed elements were labeled to describe their content (e.g. ‘I put this on the scale of make sure I don’t eat too much’ was labeled as ‘calculating/weighing food’). In the third phase, the codes were assigned to the priorly constructed seven thematic categories from the quantitative analysis (e.g. the example above was assigned into the third category of body control). Step four involved reviewing and checking if the themes are fitting the data, followed by the definition and naming of added themes (step five). When the five steps were complete, the coding process and formation of the thematic clusters were discussed and reviewed by peers.

A common shortcoming of thematic analyses on YouTube videos are that visual content is easily neglected. Therefore, the first author additionally analyzed visual representations such as facial expressions and body movements.

## 3 Results

The results from the quantitative content analysis and the thematic content analysis show us two important things. First, energy balance related behavior (EBRB, food and physical activity in terms of calorie intake and expenditure) is the central theme in the vlogs coming from 2019. Second, these themes are much less popular in 2020 and instead the concept intuitive eating comes to the foreground. An EBRB index variable was formed based on the codes: calling a product high calorie, hesitating to consume a product because it is high in calories, negative comments about the body shape and compensating in the food intake.

### 3.1 Dieting and intuitive eating

As reflected in Table 1, the codes from the EBRB index variable are averagely being mentioned 3.5 times per video in 2019, but only 0.5 times in 2020. The same goes for the usage of ‘MyFitnesssPal’, which is a calorie intake tracking app. The app is used and mentioned 0.50 times per video in 2019, contrasting only 0.14 times in 2020. Also, simply mentioning the word 'calorie' occurs more in the video’s originating from 2019, namely 3.6 times per video, contrasting 0.5 times in 2020. All these results are significant and point in the same direction.

**Table 1:** T-tests comparing pre- and during COVID-19 themes.

	N	Mean 2019	N	Mean 2020	Sig. T-test
*IndexEBRB*	16	3.4375	21	0.5238	0.001
*MyFitnessPal*	16	0.50	21	0.1429	0.018
*Calories*	16	3.6250	21	0.5238	0.012
*Eating what I want to*	16	0.3125	21	1.00	0.016
Intuitive eating	16	0.4375	21	1.00	0.103

These results matched the results from the qualitative analysis. Again, counting calories, losing weight and the app ‘MyFitnessPal’ were core themes throughout the vlogs, structuring their narrative.

Vlogger Milou mentioned in one of her vlogs:

“Allright, so I calculated: 20 g of cheese. I know it’s not a lot, but cheese has a lot of calories that can accumulate quickly and I don’t want to put that on my pizza.”

This phrase could be classified within the sphere of ‘wellness diets’ where the idea is evoked that an ideal of optimal health can be achieved through the correct diet [14].

The fact that vlogs during COVID are less concerned with calories raises the question what is mentioned instead. Our results show that the usage of the concept ‘intuitive eating’ was used more in 2020: 0.44 times in 2019 compared to 1.0 time per vlog in 2020. The same effect can be found in phrases where vloggers express that they eat whatever they want to. As can be observed in Table 1, it’s mentioned averagely 0.31 times per video in 2019, compared to 1 time per video in 2020.

These differences were also shown amongst the qualitative content analysis. Vlogger Milou tells her viewers:

“I’m trying to listen to my body more and more. I try not to prepare myself too much food. If I’m hungry later, I will just make myself some more.”

### 3.2 Claims of micro nutritional value

Looking at the results of the averages vloggers talk about avoiding or taking products because of their nutritional value, a few things can be said. Firstly, the importance of protein. Protein and protein containing products are, as reflected in Table 2, averagely mentioned 2 times per video in 2019 compared to 0.90 times in 2020. Even though there is an observable decline, protein and protein containing products are still mentioned in almost every vlog. Health claims about carbs and fat were only found when talking about them in a negative sense: avoiding products who are high carb or high fat. Calling products high carb happens slightly less in 2020.

**Table 2:** Nutritional and health claims.

	N	Mean 2019	N	Mean 2020	Sig. T-Test
Indexprotein	16	2	21	0.9048	0.068
Indexhighcarbs	16	0.5625	21	0.1905	0.139
Controle: avoid fatty foods	16	0.00	21	0.0476	0.390
Healthfoods	16	2.8125	21	5.6190	0,001

### 3.3 From dieting to food freedom?

The vloggers in our study move from counting calories to intuitive eating. But, this trend does not mean a decline in healthy foods or more vlogs filled with junk food in 2020. Contrarily, healthy products are more displayed in the vlogs from 2020, as reflected in Table 2. During this research, the most consumed ‘health’ foods were counted and combined in the index variable ‘Healthfoods’. This includes salads, avocado, smoothies, peanut butter, oatmeal, ginger tea, extra vegetables, and lemon water. As reflected in table 2, we see that healthfoods were mentioned twice as much during the COVID-19 period.

## 4 Discussion and conclusion

There is ample evidence of changes in body weight, food and supplement intake, alcohol consumption and physical activity during the COVID-19 pandemic. However, even on a cross-country aggregate level, we see diverging results: everyday habits became partly healthier and partly unhealthier [[1], [2], [3], [4], [5], [6], [7], [8], [9], [10]]. Current reviews seem to suggest that these effects are specific for gender, age, health status, prior habits, education and country context at least. In this research, we have therefore focused on a particular country, the Netherlands, and the online food culture within it. This allows us to get a closer look at changes during pre-post COVID-19.

Looking at changes in the Dutch online foodscape through the lens of Crawford’s dimensions of healthism [17,18], we witness that from 2019 to 2020, “body control” seemingly relaxes to some degree and “health claims” focusing on micronutrients are less frequent. However, displaying and discussing healthy food is even more present in 2020 Dutch food-vlogs. In that sense, health as a core ideology is maintained.

We also see a shift from counting calories, restricting intake and burning calories through exercise to intuitive eating during COVID-19. Intuitive eating grew in popularity as an ‘anti-dieting’ claim [27,28]. However, we suggest that intuitive eating might be a new way of dieting. Relaxing food restrictions may avoid cravings and binges associated with other diets. Rather than seeing the shift towards intuitive eating as the loosening of “body control” in the sense of Crawford [17], we might also think of it as a more subtle form of control: carefully letting go of restrictions and obtaining some food freedom as a way to be in control of cravings and binging. Potentially, intuitive eating provides a legitimation and control option for those who cannot fully adhere to dieting, or those who feel dieting is not morally righteous. This shift in control could be related to the restrictions experienced during the COVID-19 pandemic. Easing food restrictions and a less restrictive diet culture might be a way to cope with the sudden (governmental) restrictions in everyday life.

We cannot ascertain here if the changes we found indeed relate to increasing bodyweight at population level as reported before [[1], [2], [3], [4]]. As our brief reference to the literature shows, we need to be specific about gender, age, country etc. since changes in habits and health are not uniform. Our contribution points to the relevance of social media [12], the prominence of “digital food cultures” [13] and in particular the role of influencers as ‘cultural intermediaries’ in the Netherlands. Rather than pointing to biopolitics in mediated foodscapes [15] in general, our study points to striking changes in frames and norms. This nuance is also relevant when approaching food vlogs and digital cultures individualizing and responsiblizing message [14]. Even within a short time frame, healthism can take different forms.

In this sense, the remarkable shift towards intuitive eating might not signal the end of diet culture. Rather, we interpret the shift towards intuitive eating as another manifestation of ‘wellness diets’ [14] which reproduces a binary moral discourse of food as ‘good’ or ‘bad’ and ‘healthy’ or ‘unhealthy’. Digital food culture, in this case Dutch vlogs, can be understood as mediated biopolitics: it strengthens the shift from professional medical authority to self-made health authorities embodying the message of self-care and of being responsible for one’s own health [18].

Taken together, although “COVID-19” was novel, the rise of intuitive eating as a newly developed healthy lifestyle in food-vlogs should be interpreted as old wine in a new bottle: a developing dieting lifestyle.

## 5 Strength and limitations

The main limitation of this study is the lack of generalizability. This is not primarily due to the size of the sample, which seems fair if one wants to ascertain the construction of meaning of these types of vlogs. However, it is unclear how the trend found in this sample relates to trends in other media or countries. Moreover, the relation between cultural constructs and actual health habits in the context of obesogenic systems [11] is beyond the reach of this article. The strength of this article is the focus on the local specificities of cultural change in media as a way to make sense of diverging outcomes of research into COVID-19 related food habits across cultures.

## Ethical standards disclosure

This research did not involve human participants and focused on publicly available vlogs.

## Data availability statement

The data associated with our study has not been deposited into a publicly available repository. However, the analyzed data consists of publicly available vlogs on YouTube. The search terms that were used for selection of the studied videos, are included in the article.

## CRediT authorship contribution statement

**Elisa Eltink:** Writing – original draft, Methodology, Investigation, Formal analysis, Data curation, Conceptualization. **Christian Bröer:** Writing – review & editing, Supervision, Conceptualization.

## Declaration of competing interest

The authors declare that they have no known competing financial interests or personal relationships that could have appeared to influence the work reported in this paper.
